RETRACTED

# Integration of Wearable Devices and English Teaching under Positive Psychology

**DOI:** 10.1155/2022/7650948

**Published:** 2022-07-19

**Authors:** Jin Zhang

**Affiliations:** School of Foreign Languages, Xinyang Agriculture and Forestry University, Xinyang 464000, Henan, China

## Abstract

Positive psychology, as a core subject to the study of people's positive power and positive quality, is intended to cultivate positive personality traits and positive emotions, and to promote the development of inspiring creativity, cooperation, and interest. The study of positive psychology provides a new perspective for our research in the field of education. The “New Curriculum Standards for Junior Middle School English” clearly states: “Students can only maintain the inner driving force of English learning and achieve results only if they have positive emotions in English learning. Negative emotions will not only affect the effect of English learning, but also affect students' long-term development. In English teaching, teachers should pay attention to students' emotions from beginning to end, and strive to create a relaxed, democratic, and harmonious teaching atmosphere. Therefore, how to infiltrate the theory of positive psychology into the frontline English teaching of junior high school becomes especially important. With the advancement of science and technology and the advent of the Internet era, various high-tech information technologies have gradually flourished, and the rapid development of information technology has promoted the reform and innovation of the teaching industry. Wearable technology is the current trend and direction of the information technology revolution. It realizes the interconnection and deep integration of people, machines and objects through the functions of collecting, sorting and analyzing mobile Internet and cloud data. The realization of wearable technology-based wearable technology not only can highly integrate educational resources, improve learning interest, but also enhance the pertinence of teaching, cultivate students' creativity, and realize personalized teaching in “full time, all-round, all fields.” This article explores the integration of wearable devices and junior high school English teaching in the context of positive psychology. First of all, this paper introduces the theoretical basis of the integration of wearable devices with English teaching. Secondly, it introduces the research methods of this paper. Finally, through questionnaires and experimental comparison analysis, it tests the interest of students in learning through the auxiliary teaching of wearable devices, and whether the academic performance has a positive effect.

RETRACTED

## 1. Introduction

With the advent of economic globalization and the age of information, English has become more and more prominent as the most important information carrier. English learning in the junior high school has a foundational value for lifelong learning and development. At the same time, the “Full-time Compulsory Education English Curriculum Standards” proposes that English learning emphasizes the importance of each student's emotions, stimulating their interest in learning English, helping them to build a sense of accomplishment and self-confidence in learning, so that they can develop a comprehensive process in the learning process. Ability to use language, improve humanities, enhance practical ability, and cultivate innovative spirit [1]. Therefore, the study of junior high school English is not only to lay the foundation for junior high school students to master a language, but also to enable students to communicate with others. More importantly, through the study of English, students can develop positive emotional attitudes, have a cross-cultural perspective, and be able to understand the country's customs and customs form a more healthy personality. Under the background of the economic era, the integration of English teaching is imperative, which provides contemporary students with rich resources for mobile learning, fully integrates modern educational technology and teaching concepts, and stimulates students' interest in learning, to improve the practical application ability of English.

However, junior high school English teaching still has excessive emphasis on grammar and vocabulary knowledge. Students' interest in English learning is not high, lack of positive English learning experience, low sense of achievement and confidence in English learning, influenced by exam-oriented education, English learning Strong utilitarianism, and other phenomena. How can we change the status quo of junior high school English teaching? This is an issue that we urgently need to solve.

The original intention of the reform is to guide college students to pay more attention to traditional culture in English learning, build college students' cultural self-confidence, correctly handle the relationship between the target language and their mother tongue, and use the springboard of language to expand language. Cultural learning vision can also make full use of cross-cultural thinking in language communication to spread mother tongue culture. This also promotes the integration of college English teaching and traditional culture, and in the actual integration, there are also some key contents that need to be paid attention to. Take this as a breakthrough for integration to ensure the effectiveness and accuracy of the integration of the two.

RETRACTED

In the 1930s, the concept of positive psychology was first proposed by two American psychologists. After a long period of development, it has attracted the attention of more and more psychologists in the world. With the continuous improvement of positive psychology theory, positive psychology has also penetrated into other fields in the continuous development, such as economics, education, and personality psychology [2, 3].

With the development of the positive psychology movement, let us re-examine the positive and negative, emphasizing that we should look at things from a positive side, not just the negative side. We should not just focus on asking questions, correcting shortcomings, but discovering advantages and make full use of advantages and promote human development. Positive psychology has been applied to politics, economics, education, and other fields and has achieved good results. Therefore, applying positive psychology to junior high school English teaching can provide a good idea for solving the problem of current junior high school English teaching [4].

Positive psychology is applied to school education and penetrates into various disciplines. It focuses on cultivating students' positive thinking ability and problem-solving ability, while at the same time focusing on the cultivation of creative thinking ability. At the same time, the concept advocated by positive psychology coincides with the basic concept of junior high school English teaching. Both advocate people-oriented, emphasize the success of experience, positive value of positive emotional experience on human development, pay attention to the emotional development of students, foster healthy personality through the cultivation of students' positive learning attitude, and stimulate interest and self-confidence.

Therefore, the application of positive psychology in junior high school English teaching has a positive impact on helping students develop positive personality, establishing a harmonious teacher-student relationship, stimulating learning English motivation and interest, and forming an active cognitive learning process. Teaching has a positive effect. Positive psychology can analyze students' attitude towards learning from psychology, and improve students' enthusiasm for learning according to the way of psychological adjustment.

In the process of applying positive psychology to English teaching, since most teachers cannot keep up with the pace of the information age, they usually use pens and rosters to record students' performance in teaching and practice, and manually analyze the weak learning of students. The link, or the simple use of information technology such as slides in the teaching process, makes positive psychology not really unfold in the process of English teaching, which limits the communication between teachers and students. Secondly, English teaching does not change the status quo of teacher teaching and student listening. Teachers do not really guide students to participate in it. Teachers are still in the center of teaching. Students can only listen to teachers, which lead to the students' main role is not good. Play it out, let alone increase students' interest in learning English, and gradually lose the role of positive psychology in education [5, 6]. In traditional teaching, teachers are responsible for teaching, students are responsible for learning, teaching is the teacher's one-way “training” activities for students, and it is manifested as: one is to teach as the centre, learning around teaching.

RETRACTED

With the advancement of science and technology and the advent of the Internet age, various high-tech information technologies have gradually flourished, and the rapid development of information technology has promoted the reform and innovation of the teaching industry [7]. Wearable technology [8] is the current trend and direction of the information technology revolution. Through the functions of collecting, sorting, and analyzing mobile Internet and cloud data, it realizes the interconnection and deep integration of people, machines, and objects. The realization of wearable technology based wearable technology [9] can not only change the current traditional teaching mode and the boring status of the English classroom, but also highly integrate educational resources, enhance learning interest, enhance teaching pertinence, and cultivate students' creativity. Achieve “full-time, all-round, all-round” personalized teaching, and learning interaction [10, 11].

Wearable device is a portable device that can be worn directly on certain parts of the human body, such as wrists, arms, or embedded in carry-on clothing and accessories. In addition to medical, military, and other special field-specific body area network sensors, with the development of sensor technology and smart chips, the popularity of civilian smart wearable devices has risen in recent years, among which Google glass and Apple watch bear the brunt, attracting research institutions and the eyes of the general public [12], the concept of smart wear is mentioned. At the same time, some smart wearables include both sensor components capable of collecting data, independent operating system and computing power, and the ability of the communication module to transmit data, and the battery life is greatly enhanced, making smart wearable equipment has become an effective way to achieve personalized teaching and zero-distance learning interaction. Wearable devices currently come in three categories: head-worn, wrist-worn, and in-wear [13, 14].

RETRACTED

In the above context, this paper explores the integration of wearable devices and junior high school English teaching, and integrates positive psychology into English teaching. First of all, this paper introduces the theoretical basis of the integration of wearable devices with English teaching; secondly, introduces the research methods of this paper; finally, through questionnaires and experimental comparative analysis [15], to understand the problems existing in current English teaching and to test wearable devices under positive psychology. Auxiliary teaching has a positive effect on students' interest in learning, English teaching participation, and academic performance. The combination of multiple theories provides the best integration scheme for the integration of English teaching, and at the same time provides a reference for the combination of wearable devices and the field of education.

## 2. Proposed Method

In the context of the information technology era, the full use of information technology, especially wearable technology, can obtain higher quality and advanced teaching resources and change the traditional English teaching mode. The effective combination of wearable technology and information teaching in the process of traditional English teaching is the only way to realize the value of positive psychology in English curriculum. In order to achieve the research goal of the integration of wearable devices and English teaching, this paper starts from the research and analysis of relevant scholars and their own teaching practice, with constructivist learning theory, mixed learning theory, humanistic theory, and multiple intelligence theory as theoretical support. In-depth integration of wearable devices with traditional English teaching and strive to explore the ideal path of traditional English teaching information is shown in Figure 1.

### 2.1. Constructivist Learning Theory

Constructivism is a study of psychology that has emerged since the mid-1980s. It is the further development of behaviorism after the development of cognitiveism, but its biggest difference from the cognitive theory of learning is that it emphasizes the initiative of learners; compared with the theory of behavior, the learning process is considered to be a qualitative change. Is an active construction process, rather than establishing a passive stimulus response model [16, 17]?

RETRACTED

There are many schools of constructivism, the most representative of which is the personal constructivism [18] proposed by American psychologist GAKelly [19], mainly von Glasersfeld [20]. The radical constructivism proposed by the representative and the social constructivism represented by Lev Vygotsky. Constructivist theory is not a specific learning theory. With the development of the times, from the objective world to subjectivism, the theory of constructivism is also in constant development [21, 22].

Constructivism believes that it is not a negative process for learners to actively acquire knowledge to learn. Therefore, teachers and learners in teaching should interact in two ways, not just the teacher. Only by adding corresponding situations to the teaching content and fully mobilizing the students' interest in learning can they truly master the corresponding skills [23, 24].

In the current traditional teaching, a piece of chalk and a book can be taught, but in the rapid development of information technology, it is obviously not advisable to be limited to the oldest traditional teaching methods. The oldest traditional teaching method is reflected in the following: (1) It is not conducive to comprehensively improving the comprehensive quality of teachers. The traditional teaching method is single, rarely involves modern teaching equipment, and relatively requires relatively high quality of teachers. It is not conducive to improving the comprehensive quality of teachers in an all-round way. (2) It is not conducive to broadening the horizons of teachers and students and expanding their knowledge. Traditional teaching does not have access to the most advanced teaching methods, such as computer networks and various audiovisual equipments. Therefore, teachers and students will only see what is in front of them, and lack understanding of the ever-changing world outside and the increasingly updated knowledge. Constructivism believes that modern multimedia is a situational creation tool and cognitive tool, such as multimedia and network, which can promote learning and facilitate communication. In teaching, the network, graphic, audio-visual, etc. can improve students' aesthetic ability, increase the technical content, enhance students' perception, and enable students to improve their interest in learning and improve the overall teaching effect.

### 2.2. Mixed Learning Theory

The hybrid learning theory combines the advantages of traditional learning methods with the advantages of wearable devices. It should not only play the leading role of teachers in guiding, inspiring and monitoring the teaching process, but also fully reflect the initiative, enthusiasm and creativity of students as the main body of the learning process. Only when time, method, learning style, and learner are appropriate, mixed learning can play its role, and its ability to deliver is appropriate. This way of learning is also optimal. This hybrid approach demonstrates the primary role of teachers and students and has become a new star in the education community. With the development of educational technology, the integration of personalized teaching into traditional teaching has gradually been recognized by the education community. Therefore, we believe that on the basis of hybrid theory learning, only by combining traditional teaching methods with individualized teaching can we truly play the leading role of students and teachers. On the one hand, taking students as the main body not only breaks the state of “teacher speaking, student listening” under the traditional learning mode, but also introduces information technology into the teaching process, fully taking into account the learners' needs, interests and hobbies, and giving them In the process of learning, they can learn knowledge and apply knowledge, cultivate their innovative ability and interest in learning, and play an important role in the future employment development of students [25]. On the other hand, the leading role of teachers in the entire teaching process cannot be ignored, because students need to apply what they have learned, the creation of situations in the teaching process, the application of wearable devices and the design of activities need teachers can complete this, and these are inseparable from the organic combination of traditional teaching and information technology. Epson released the Pulsense series of wearable devices, including smart watches and smart bracelets. These products integrate Epson's industry-leading original biosensing technology and cloud-based system services to meet the fitness, health, and fitness needs of the wearable consumer goods market and exercise needs.

RETRACTED

### 2.3. Humanistic Learning Theory

Humanistic learning theory focuses on the teaching process rather than the teaching content. It is a teaching method rather than a teaching effect. It focuses on how to create a good learning environment, allowing learners to view the world from their own perspective, understand the world, and achieve the highest level of self-realization. According to Rogers, human beings have natural learning aspirations and potentials that can be released under appropriate conditions; the goal of teaching is to promote learning, which should be driven by curiosity, and students consciously absorb any knowledge of interest and need; the task of the teacher. It is not to teach students to learn knowledge, nor to teach students how to learn [26]. Contrary to this, it provides learners with a wealth of learning resources, builds an atmosphere conducive to learning, and allows learners to decide how to learn.

Under the guidance of this idea, American scholars put forward the study and teaching concept of “free learning” and “student center” in the 1960s. He emphasized that teaching should cultivate students' individuality, fully mobilize the internal motivation of students' learning, and create a harmonious teaching [27]. However, traditional education is more like a kind of machine production education. There is no individuality, no soil for personality development, more like a factory, mechanically producing batches of products, and expect the same type of products to be exactly the same.

The wisdom teaching assisted by wearable technology reflects this theory. Teachers collect a large amount of student data through wearable devices, and accurately analyze students' individualized learning needs, learning content, learning process, learning progress, and data through data. Learning strategies, learning activities, learning methods, learning evaluation, and other characteristics, and accordingly develop corresponding teaching plans, truly teach students in accordance with their aptitude, truly realize humanistic learning, maximize the development and development of each student's personal expertise, and thus subtly influence students' learn in depth and learn smartly.

### 2.4. Multiple Intelligence Theory

The theory of multiple intelligence is a reform trend that swept the American education community in the 1980s, presented by Howard Gardner. Gardner and his theory of multiple intelligences believe that in addition to language intelligence and mathematical logic intelligence, there are at least six other kinds of intelligence: “space intelligence,” “body movement intelligence,” “music intelligence,” “interpersonal intelligence,” “Introspective Intelligence,” and “Nature Observation Intelligence” have since added “existence of intelligence.” According to Gardner, intelligence is multiple, with at least seven intelligences and eight known intelligences in each person. The theory of multiple intelligences believes that different people have different cognitive strengths and corresponding cognitive styles, with particular emphasis on each person's own way of understanding knowledge and constructing their own understanding of things [28].

In the process of deep integration of wearable devices and English teaching, teachers must first become “multi-intelligent” teachers, but also pay attention to the comprehensive and coordinated development of students. When arranging teaching activities, we should use information technology, take into account the learning content in the field of multiple intelligences, and fully apply diversified teaching methods. At the same time, we provide learning activities that are conducive to the development of multiple intelligences, and establish multiple evaluation criteria to develop each student's multiple intelligences.

RETRACTED

## 3. Research Method

By paying attention to the research dynamics of positive psychology at home and abroad, we find out the shortcomings of junior high school English teaching, which is taken as the research value and the innovation of research. Questionnaire survey was conducted on 240 students in the school, and they went deep into the specific environment of junior high school teaching. They conducted on-the-spot observations on teachers, students, and the environment. Afterwards, they used four classes, one class and three classes. The wearable equipment experimental class, the second class, and the fourth class are traditional teaching classes. In the experimental process of the different teaching modes of the four classes in one academic year, the comparative analysis of the results and the classroom state is carried out to verify the wearable devices based on positive psychology.

### 3.1. Questionnaire

In order to understand the attitudes and interests of junior high school students in English learning and the willingness to participate in English classes, and to understand the impact of school learning environmental factors on English learning, this paper refers to other researchers' questionnaires and combines their own teaching. The experience and the positive factors of positive emotion, positive personality, and positive environment in positive psychology compiled the “Question Questionnaire for Junior Middle School English Teaching Status.” The questionnaire has three dimensions.

  Dimension 1: Positive emotions: Junior high school students' attitudes and interests in learning English.
  Dimension 2: Positive personality: the participation of junior high school students in the English class; the evaluation method adopted by the junior middle school English teacher.
  Dimension 3: Positive environment: Environmental factors that affect junior high school English learning.

On the basis of the “Questionnaire on the Present Situation of Junior Middle School English Teaching,” in order to verify whether the wearable device helps English teaching in the middle school English classroom teaching, whether it has effect on the positive emotions and positive personality cultivation of students, and demonstrate its feasibility, this paper has also compiled “Questionnaire for the teaching of wearable equipment for junior high school English classrooms,” the questionnaire surveyed 240 students in the four classes taught by the students. The method of questionnaire distribution was mainly on-site, on-site recycling to ensure the recovery rate.

RETRACTED

### 3.2. Experimental Comparison

This study adopts the method of natural experiment, which is a method of creating and controlling certain conditions for research under the conditions of daily teaching. The teacher in the class is the same person, and the teaching materials are the same, and the teacher environment is the same. The experimental subjects of this study are the four classes taught by them. Two are experimental classes using wearable device teaching, and the other two are traditional teaching classes. The experimental environment is a real classroom teaching environment. The object to be tested was purposely observed before and during the experiment.

In the daily teaching, the teaching design practice in the wearable device environment is carried out at the same time, and the teaching strategy of positive psychology is actively adopted. It is applied to classroom teaching and infiltration after class, and forms a positive teaching style in continuous practice. The effectiveness of wearable devices based on positive psychology in junior high school English classroom teaching is verified by the results of four experimental classes, the state performance of students in class, and the overall learning atmosphere of the class.

## 4. Research Results and Analysis

### 4.1. Questionnaire Results

The “Secondary English Teaching Status Questionnaire” dimension is a positive emotion. It is mainly for students' attitudes and interests in junior high school English learning. The test results are shown in Table 1. After that, the junior high school is conducted for one class and three classes. The questionnaire of the English classroom wearable device assisted teaching compares and analyzes the improvement of the interest of students in learning English by integrating wearable devices into English teaching. The comparison results are shown in Figures 2 and 3.

It can be seen from the data in Table 1 that under the traditional teaching mode, 240 students from four classes are very interested in English, accounting for 27.9%, 31.7% are interested, and 40.4% are interested in learning English. From the data in Figures 2 and 3, by applying wearable devices to English classroom teaching, the interest in learning for one class and three classes has been greatly improved. A class of students who are very interested in English has 33 students, accounting for 55%, 18 students are interested, accounting for 30%, and the proportion of students with higher learning interest is 20% higher than traditional teaching; The number of students who are very interested in English is 32, accounting for 53.3%, 17 students are interested, accounting for 28.3%, and the proportion of students with higher learning interest is 21.6% higher than traditional teaching. The combination of wearable devices and junior high school English teaching has an obvious effect on the improvement of students' interest in learning.

RETRACTED

In the second dimension of positive personality, the test is mainly for the participation in the student learning. The test results are shown in Table 2. By applying the wearable device to the English classroom teaching, the participation of the class activities of the four classes is compared. The comparison results are shown in Table 3 and Figure 4.

It can be seen from the data in Table 2 that under the traditional teaching mode, 240 students from four classes in the English course actively participated in 27.9% of the students, and occasionally participated in the student accounted for 31.7%. According to the data in Table 3, by integrating wearable devices with English classroom teaching, the proportion of students actively participating in the curriculum reached 46.3%, which was 19% higher than before, and the proportion of passive participation and nonparticipation. The ratio was 26.6%, which was 13.8% lower than before. From the data analysis of Figure 4, the number of active participants in the experimental class was far more than that in the traditional class. The proportion of active participants in the course reached 65.8%. The integration of junior high school English teaching has a positive effect on students' active participation in the teaching of the subject.

In the three dimensions of positive environment, the impact on student learning is mainly explored from the perspective of learning environment. The test results are shown in Table 4.

From the data in Table 4, it can be seen that the teacher encourages the highest proportion of the way to promote English learning, reaching 39.2%. Parents and friends encourage 30.4% and 28.3%, respectively, and the parents of parents are the least concerned, accounting for 2.1%. The above data shows that the teacher plays an important role in the students' minds, and the students on the four levels hope to be encouraged by the teacher. The encouragement of parents and friends is also very important. Therefore, it is crucial for students to learn, build a positive environment, and support students to encourage and influence students' learning. Therefore, the integration of wearable devices with English teaching can enable teachers, parents, and friends to promptly and effectively encourage students. The integration of wearable devices into English language teaching allows for a greater variety of forms of English language teaching, as well as providing an environment for students to express themselves and breaking down the limitations of existing teaching, such as the ability to gather in a classroom and the inconvenience of dictation.

RETRACTED

### 4.2. Experimental Results and Discussion

In the context of positive psychology, wearable devices have a positive effect on the improvement of students' English academic performance in English classroom teaching. In this paper, the final grades of two semesters of four courses were tested, and the results are shown in Tables 5 and 6.

As can be seen from the above two tables, after one year of experiments on the integration of wearable devices with English teaching, the experimental class using wearable device teaching has significantly improved academic performance. After the first semester of the 2015–2016 school year, wearable equipment was applied to English teaching. The average scores of one class and three classes of English reached 92 points or more, which was more than 10 points higher than the average scores of the second and fourth classes of traditional teaching. In terms of rate, the experimental class is 9 percentage points higher than the traditional teaching class; in terms of pass rate, the experimental class is more than 85%, which is higher than the traditional teaching class by more than 20 percentage points. After the application of the second semester, the overall performance of the experimental class has been significantly improved. The average score of one class is 97.5, the average of three classes is 96.6, the rate of excellence is over 50%, and the pass rate is over 95%. In contrast to traditional teaching classes, the overall score has hardly improved, but has declined.

Through the in-depth teaching of information technology, students' interest and enthusiasm for learning English have been greatly improved, and the initiative of learning has been greatly improved. The students who have no interest in the words are reminiscent of the taste of wearable devices and between students. The competition of the leaderboards has become willing to memorize words, and dictation scores have passed from pass to pass, and then to good; students who are not willing to communicate with teachers can be discussed with teachers and classmates through time and space through wearable devices. This increases self-confidence and also asks teachers to exchange questions after class, which is beneficial for teachers to accurately analyze students and conduct precise counseling. It can be seen that compared with traditional teaching, the teaching performance techniques assisted by wearable devices are more diverse, three-dimensional and vivid, the teaching resources are more abundant, the learning time is more flexible, the limitations of teacher-student communication are better solved, and the teachers and students are improved. The interaction between students and students is more effective in improving students' academic level.

RETRACTED

Teaching the same content in four classes, the experimental class uses the learning platform carried by the wearable device, and adopts the information-assisted teaching method. The space and time of teaching are flexible. As long as the Internet is convenient, students can learn, discuss, and Questioning, doing homework and testing, teachers can track the whole process of student learning anytime, anywhere, online answering, correcting homework, etc., to understand the progress and quality of students and knowledge and skills. The network of teaching resources in the era of “Internet +” not only greatly reduced the teaching burden for teachers, but also made students enjoy the convenience of learning. After the lecture, the students in the experimental class generally reflected that the teaching method is easy to understand and not boring. Knowledge is also more solid, and there are automatically generated sets of wrong questions, all of which have generated a strong interest in the students from the beginning.

## 5. Conclusion

After decades of research and development, positive psychology aims to cultivate positive personality traits and positive emotions. The concept of inspiring creativity, cooperation spirit, and interest development has been deeply rooted in people's minds, and its application range is increasing widely. The research of positive psychology provides a new perspective for the research in the field of education. How to infiltrate the positive emotions, positive personality and positive environment of positive psychology into the frontline teaching is particularly important. With the advancement of science and technology and the advent of the Internet age, the rapid development of information technology, traditional classroom teaching, and information technology is equivalent to the two wings of education; only two wings cooperate with each other, at the same time function, a new hybrid. The teaching model can soar in the blue sky of education and bring about the spring of educational reform. In this context, this paper explores the integration of wearable devices with junior high school English teaching. First of all, this paper introduces the theoretical basis of the integration of wearable devices with English teaching. Secondly, it introduces the research methods of this paper. Finally, through questionnaires and experimental comparison analysis, it tests the interest of students in learning through the auxiliary teaching of wearable devices, and whether the academic performance has a positive effect. The research results confirm that junior high school English teaching assisted by wearable devices not only can highly integrate educational resources, improve learning interest, but also realize “full-time, all-round, all-field” personalized teaching and learning interaction, and improve students' classroom participation and academic achievement.

RETRACTED

## Figures and Tables

**Figure 1:** Theoretical framework.

**Figure 2:** Comparison of English learning interest of class 1 students.

**Figure 3:** Comparison of English learning interest of class 3 students.

**Figure 4:** Comparison of the participation of wearable devices in the English teaching classroom.

**Table 1:** Four classes of students' interest in English learning (person).

Questionnaire results	Class 1	Class 2	Class 3	Class 4	Percentage (%)
Very interested	18	16	17	16	27.9
More interested	21	18	19	18	31.7
Not interested	14	16	13	14	23.8
Not interested at all	7	10	11	12	16.6

**Table 2:** Participation in the English class activities of four class students (person).

Questionnaire results	Class 1	Class 2	Class 3	Class 4	Percentage (%)
Active participation	18	15	17	17	27.9
Occasional participation	21	19	19	17	31.7
Passive participation	14	16	13	14	23.8
Give up participation	7	10	11	12	16.6

**Table 3:** Participation in activities after the integration of wearable devices and English teaching (person).

Questionnaire results	Class 1	Class 2	Class 3	Class 4	Percentage (%)
Active participation	41	15	38	17	46.3
Occasional participation	14	19	15	17	27.1
Passive participation	3	16	5	14	15.8
Give up participation	2	10	2	12	10.8

**Table 4:** Ways to promote English learning (person).

Questionnaire results	Class 1	Class 2	Class 3	Class 4	Percentage (%)
Teacher encourages	24	25	22	23	39.2
Parental encouragement	20	18	16	19	30.4
Friend encouragement	15	16	19	18	28.3
Teacher and parents indifferent	1	1	3	0	2.1

**Table 5:** Analysis of the final exam results of the first semester of the 2015–2016 school year.

Class		Class 1	Class 2	Class 3	Class 4
Student population		60	60	60	60
English scores	Average	93.4	81.6	92.3	82.1
	Excellent rate (%)	29.6	20.6	30.1	22.3
	Pass rate (%)	85.3	61.7	87.3	64.3

RETRACTED

**Table 6:** Analysis of the final exam results of the second semester of the 2015–2016 school year.

Class		Class 1	Class 2	Class 3	Class 4
Student population		60	60	60	60
English scores	Average	97.5	82.5	96.6	81.8
	Excellent rate (%)	51.2	21.3	50.3	21.7
	Pass rate (%)	97.6	62.3	96.8	62.8

## Data Availability

The data that support the findings of this study are available from the corresponding author upon reasonable request.
